The article "The Levels of TNF-α, Tissue Factor, and Coagulation Function in Rats with Pulmonary Hypertension and the Intervention Effect of Sildenafil Encapsulated by Targeted Nanocarriers" was retracted in 2023. Reasons: unreliable results or conclusions; concerns about the data; concerns about the peer review; concerns about the citations.

# The Levels of TNF-*α*, Tissue Factor, and Coagulation Function in Rats with Pulmonary Hypertension and the Intervention Effect of Sildenafil Encapsulated by Targeted Nanocarriers

**DOI:** 10.1155/2022/8619092

**Published:** 2022-05-13

**Authors:** Xuan Ma, Xue-E Wang, Lin-Xia Xie, Sha Lu, Cheng Jiang

**Affiliations:** ^1^Department of Respiratory Medicine, Xi'an International Medical Center Hospital, Xi'an, 710100 Shaanxi, China; ^2^Department of Pulmonary and Critical Care Medicine, Sleep Disease Medical Center, The Affiliated Hospital of Jianghan University, Wuhan, 430000 Hubei, China

## Abstract

Pulmonary hypertension (PAH) is a proliferative disease of pulmonary blood vessels, but the pathogenesis of pulmonary hypertension is still unclear. This article explores the role of tumor necrosis factor-*α* (TNF-*α*), tissue factor (TF), and coagulation function (CF) in the pathogenesis of PAH. PAH is often accompanied by vascular intima injury and muscular arterial media thickening. Coupled with the wide application of nanotargeted drugs in recent years, a targeted nanocarrier encapsulating sildenafil was prepared in this study. The particle size, PDI, zeta potential, drug loading, and encapsulation efficiency were 194.32 ± 17.31 nm, 0.28 ± 0.02, −6.34 ± 0.33, 24.61%, and 70.52%. The monocrotaline PAH rat model was constructed, and it was found that the levels of TNF-*α*, TF, and CF in the peripheral blood of PAH rats were abnormally increased. 30 PAH rats were randomly divided into 5 groups and injected with saline (NS group), sildenafil (sildenafil group), target the nanoempty carrier (TNC-E group), ordinary nanocarrier encapsulated sildenafil (CNC-sildenafil group), and targeted nanocarrier encapsulate sildenafil (TNC-sildenafil group). Compared with the NS group, the mean pulmonary artery pressure in the TNC-sildenafil group was lower (*P* < 0.05). Compared with the normal rat group, the pulmonary small blood vessel media thickness, TNF-*α* level, TF level, and the area of myocardial cells were increased in the NS group, sildenafil group, TNC-E group, and CNC-sildenafil group (*P* < 0.05). Compared with the NS group, the pulmonary small blood vessel media thickness, myocardial cell area, and the levels of TNF-*α* and TF in the TNC-sildenafil group were reduced (*P* < 0.05). Targeting nanocarrier encapsulation of sildenafil can obviously reduce the average pulmonary artery pressure in rats with pulmonary hypertension, improve pulmonary vascular media proliferation and myocardial hypertrophy, and restore the levels of TNF-*α*, TF, and CF to a normal state.

## 1. Introduction

Pulmonary arterial hypertension (PAH) is a disease in which the pulmonary arteries are abnormally elevated due to some reasons. The main clinical symptoms are abnormal shortness of breath, accompanied by chest tightness, dizziness, fatigue, and other symptoms. The onset of PAH in children may lead to developmental delay or abnormality, which is not conducive to the physical and mental health of patients [1, 2]. The main causes of PAH are heart disease, autoimmune disease, blood disease, genetic mutations, etc. that lead to vasoconstriction, pulmonary artery wall remodeling, and in situ thrombosis, which in turn increases pulmonary vascular resistance [3–6]. However, PAH has a wide range of causes, and the pathogenesis of PAH has not yet been fully clarified. Studies have found that changes in coagulation function play an important role in the occurrence and development of PAH [7]. Inflammatory factors may play a dominant role in the changes of coagulation function [8]. Therefore, this article discusses the role of tumor necrosis factor-*α* (TNF-*α*), tissue factor (TF), and coagulation function (CF) in the pathogenesis of PAH and provides guidance for the prevention and treatment of PAH.

The article "The Levels of TNF-α, Tissue Factor, and Coagulation Function in Rats with Pulmonary Hypertension and the Intervention Effect of Sildenafil Encapsulated by Targeted Nanocarriers" was retracted in 2023. Reasons: unreliable results or conclusions; concerns about the data; concerns about the peer review; concerns about the citations.

PAH is a proliferative disease of pulmonary blood vessels, often accompanied by vascular intima injury and muscular arterial media thickening, which in turn causes luminal stenosis and decreased elasticity. As the disease progresses, it will eventually lead to right heart failure [9] . How to inhibit the excessive proliferation of pulmonary vascular media smooth muscle cells and promote cell apoptosis is the key to reversing pulmonary vascular disease. The current clinical treatment of PAH drugs include sildenafil and prostacyclin. Although these drugs can expand the pulmonary artery, inhibit the proliferation of pulmonary vascular media smooth muscle cells and promote apoptosis, and alleviate vascular inflammation to a certain extent, they cannot improve the patient's activity endurance and long-term survival rate. It may be closely related to the inability of the drug to reach an effective therapeutic concentration in the damaged blood vessel of the lung tissue [10, 11]. In recent years, targeted nanomaterial-encapsulated drugs have been widely used in the field of biomedicine, especially in antitumor therapy. By designing the ligands of the characteristic molecules of tumor cells on the surface of the nanoparticles, the specific binding between the nanoparticles and the tumor cells is promoted. In order to achieve targeted therapy of tumors, increase the concentration of drugs in the target area, thereby improving the utilization and efficacy of drugs and reducing adverse drug reactions [12, 13]. Studies have shown that the PAH model pulmonary arteriole media smooth muscle cell surface glucose transporter-1 (GLUT-1) is highly expressed, aerobic glycolysis is enhanced, and 18 fluorodeoxyglucose (18F-FDG) uptake is increased [14]. To improve the effectiveness and targeting of sildenafil, based on the above theory, this experiment designed a targeted drug targeting the GLUT-1 site on the surface of smooth muscle cells in the pulmonary arteriole media, that is, a glucose-modified nanocarrier encapsulating sildenafil and targeted binding to the diseased pulmonary blood vessels. It is the first time to observe the therapeutic effect on pulmonary arterial pressure and pulmonary vascular injury in rats with PAH, aiming to provide new guidance and suggestions for the treatment of PAH.

The article "The Levels of TNF-α, Tissue Factor, and Coagulation Function in Rats with Pulmonary Hypertension and the Intervention Effect of Sildenafil Encapsulated by Targeted Nanocarriers" was retracted in 2023. Reasons: unreliable results or conclusions; concerns about the data; concerns about the peer review; concerns about the citations.

## 2. Materials and Methods

### 2.1. Experimental Materials and Grouping

36 male SD rats, 2 months old, weighing 210 g ± 5 g, were purchased from Nanjing Junke Biological Engineering Co., Ltd. The rats all drink and eat freely. Six rats were randomly selected as the normal control group, and the remaining 30 rats were used to construct the PAH model. The monocrotaline (Item No: C2401; Sigma-Aldrich) solution 60 mg/kg [15] was subcutaneously injected into the neck back of 30 rats. Average pulmonary arterial pressure (mPAP) ≥ 25 mmHg detected by right jugular vein catheterization in rats was regarded as successful pulmonary arterial hypertension model. After 4 weeks, 30 PAH model rats were randomly divided into 5 groups. Five groups of rats were injected with 8 mg/kg sildenafil (sildenafil group; Pfizer, China), targeted nanoempty carrier (TNC-E group), ordinary nanocarrier encapsulated sildenafil (including sildenafil 8 mg/kg, CNC-sildenafil group), targeted nanocarrier encapsulated sildenafil (including sildenafil 8 mg/kg and TNC-sildenafil group), and equal volume of normal saline (NS group); once a day, continue to inject for 2 weeks. All operations and animal handling follow the laboratory animal guidelines and animal experiment ethics formulated by the national health agency. The use of laboratory animals strictly abides by the regulations on the protection and use of hospital animal experiments.

### 2.2. Preparation of Targeted Nanocarriers to Encapsulate Sildenafil

0.5 g of lactide glycolide copolymer 50 : 50 (PLGA, Boehringer Ingelheim) was dissolved in 10 mL of anhydrous dimethylformamide (DMF). And 0.05 g of N-hydroxysuccinimide (NHS, Sigma-Aldrich) was added to the PLGA solution. After 1 h, add dicyclohexylcarbodiimide (DCC, Sigma-Aldrich) and continue stirring for 2 h. The precipitated polymer was dried under vacuum and stored at -20°C. The obtained polymer was further dissolved in DMF and mixed with 0.5 mL glucosamine solution (0.02 g dissolved in 0.5 mL distilled water) and reacted on an ice bath for 3 h. Pour the modified polymer into 100 mL of distilled water to precipitate. The precipitated polymer was filtered and dried under vacuum to obtain a glucose-PLGA polymer, which was stored at -20°C.

The article "The Levels of TNF-α, Tissue Factor, and Coagulation Function in Rats with Pulmonary Hypertension and the Intervention Effect of Sildenafil Encapsulated by Targeted Nanocarriers" was retracted in 2023. Reasons: unreliable results or conclusions; concerns about the data; concerns about the peer review; concerns about the citations.

Preparation of glucose-PLGA nanoparticles containing sildenafil was as follows: 150 mg glucose-PLGA was dissolved in 10 mL ethyl acetate to obtain an organic solution. 25 mg of sildenafil was dissolved in 2 mL of 0.3% F-68 aqueous solution to obtain a water system. The ultrasonic power is 30%, and the intermittent ultrasonic is 60 s. The water system was dispersed in the organic solution to form colostrum. 3 mL of colostrum system was placed in 9 mL of 0.05% F-68 aqueous solution for ultrasound. The ultrasonic power is 30%, and the intermittent ultrasound is 60 s to form a double emulsion system. The double emulsion was poured into a 90% ethanol solution and stirred magnetically for 40 min. The resulting nanoparticle suspension was placed in a dialysis bag with a molecular weight cut-off of 24 k. The dialysis bag was placed in 1.8 L of deionized water for 2 hours and then dialyzed three times. Finally, the obtained system is frozen and then placed in a freeze dryer for freeze drying to obtain drug-loaded nanoparticles.

Nanoparticle size, PDI, and zeta potential measurement were as follows: 50 mg of nanoparticle freeze-dried powder was ultrasonically dispersed in distilled water. Suspension is sucked by a dropper and dropped into a quartz cuvette. The particle size, PDI, and zeta potential of the nanoparticles were measured with a nanoparticle size and zeta potential analyzer (Malvern, Britain). Observe the nanoparticles through a transmission electron microscope (HITACHI, Japan).

Determination of drug loading of nanoparticles was as follows: 30 mg of glucose-PLGA lyophilized nanoparticles containing sildenafil was fully dissolved in 3 mL of DMSO to form a solution. An ultraviolet-visible spectrophotometer UV3600 (absorption wavelength of 390 nm; Shimadzu, Japan) was used to test the absorbance of the sample. Calculate the mass of sildenafil contained in the nanoparticles according to the “sildenafil-DMSO standard curve equation.” Calculate the drug loading of nanoparticles according to the formula: actual drug loading = drug mass in lyophilized powder/total mass of recovered lyophilized powder∗100%:

(1) $$\begin{array}{c} \text{Theoretical drug loading}=\text{drug dose}/\left(\text{drug dose}+\text{nanoparticle matrix quality}\right)*100\%. \end{array}$$

### 2.3. In Vitro Drug Release Experiment of Drug-Loaded Nanoparticles

The sustained-release effect of nanoparticles under different pH conditions was observed to evaluate the structural stability and sustained-release properties of drug-loaded nanoparticles. A certain concentration of drug-loaded nanoparticle solution was placed in a dialysis bag (Sigma, USA). After sealing the dialysis bag with a dialysis clip, put it into a brown reaction flask containing different pH release media (PBS, pH 4.6, pH 7.4) and oscillate (100 r/min) in a constant temperature water bath at 37°C for 72 h dialysis. A certain volume of dialysate was taken out of the brown reaction flask at regular intervals. The absorbance value was measured at 480 nm by an ultraviolet spectrophotometer, and an equal volume of the corresponding buffer was added to the reaction flask at the same time. Calculate the cumulative release percentage of sildenafil in different release systems according to the standard curve of sildenafil and draw the release curve.

The article "The Levels of TNF-α, Tissue Factor, and Coagulation Function in Rats with Pulmonary Hypertension and the Intervention Effect of Sildenafil Encapsulated by Targeted Nanocarriers" was retracted in 2023. Reasons: unreliable results or conclusions; concerns about the data; concerns about the peer review; concerns about the citations.

### 2.4. Pulmonary Arterial Pressure Measurement

The rats were anesthetized by intraperitoneal injection of ketamine hydrochloride 100 mg/kg (Shandong Fangming Pharmaceutical Group Co., Ltd., China) and fixed on the rat board in the supine position. The rat's tongue was wrapped with gauze, and the tongue was slightly pulled to expose its glottis. Wipe the secretions on the oral surface with a wet cotton swab. Insert a 16# trocar through the mouth, connect to the ventilator, and set the breathing rate to 60 beats/min. One end of the tracheal tube was fixed to the neck skin of the rat, and the other end was properly connected and fixed with the breathing circuit pipeline. Iodine disinfection, after preparing the skin, enter the chest at the strongest heartbeat, cut off two or three ribs and ligate, cut a happy bag, and stuff it with small gauze. The 24# indwelling needle punctures the right ventricular outflow tract and inserts the overtube into the main pulmonary artery and connects the pressure transducer to the other end. When the pulmonary artery pressure waveform appears on the monitor screen of the ECG monitor (Felles Photonic Instruments, China) and was stable for 1 minute, record the pulmonary artery pressure value at this time.

### 2.5. Detection of TNF-*α*, TF, and CF in Peripheral Blood

The femoral artery was cut in the left groin of the rats, and 3 ml blood was taken in a clean test tube. The blood was centrifuged at 1500 rpm for 5 min in a normal test tube, and the serum was collected. The ELISA method was used to detect the levels of TNF-*α* and TF in the peripheral blood of rats. After the rats were anesthetized in the abdominal cavity, 4 mL of blood was collected from the abdominal aorta in a vacuum tube and centrifuged at 3000 r/min for 5 min. After taking the upper layer of serum, it was stored at -80°C ultra-low temperature for testing. The test was performed in strict accordance with the ELISA kit instructions (Beyotime, China), and the brief steps were as follows: (1) dilute the specimen and washing solution, (2) set the standard product, (3) add sample and incubate, (4) add the first antibody incubation, (5) add enzyme labeling work (6), incubation with substrate working solution, and (7) stop and measure the absorbance (*A*) value.

The article "The Levels of TNF-α, Tissue Factor, and Coagulation Function in Rats with Pulmonary Hypertension and the Intervention Effect of Sildenafil Encapsulated by Targeted Nanocarriers" was retracted in 2023. Reasons: unreliable results or conclusions; concerns about the data; concerns about the peer review; concerns about the citations.

After the rat was anesthetized, 3 ml of abdominal aortic blood was placed in a trisodium citrate blood collection tube. The CF indexes of the automatic coagulometer include prothrombin time (PT), thrombin time (TT), and fibrinogen (FIB).

### 2.6. Measurement of the Media Thickness of Small Pulmonary Vessels and the Area of Myocardial Cells

The infusion thong was connected to the indwelling needle, the red blood cells in the pulmonary blood vessels were washed with normal saline, and the left atrial appendage was cut open until the heart and lung tissues become white. The animals were killed by injecting 5 mL of 10% potassium chloride (Solebo, China) through the pulmonary artery. Then, 10% paraformaldehyde (Solebo, China) was perfused through the tracheal tube. After the lung tissue was uniformly expanded for 5 min, the left and right ventricles and the right lower lung tissue were removed and fixed.

Pulmonary vascular morphology detection was as follows: the lung tissue was paraffin-embedded and sectioned with HE staining. The small pulmonary blood vessels were observed and photographed under an electron microscope. There were 3 specimens in each group and 5 blood vessels in each specimen. The diameter of the media (the thickness MT between the inner and outer elastic plates) of the pulmonary arterioles (50-150 *μ*m in diameter) and the diameter ED between the outer elastic plates were measured with Image-Pro Plus6.0 software. Calculate the media thickness (WT) = (2MT/ED) × 100%.

Measurement of myocardial cell area was as follows: after HE staining of the right ventricle, 3 specimens were selected from each group. Each specimen was selected 20 right ventricular cardiomyocytes, circled the cardiomyocyte boundary, and calculated its area (*μ*m^2^) through OLYMPUS cellsens Dimension software.

### 2.7. Statistical Analysis

SPSS23.0 software was used to analyze the data. Normally distributed measurement data are expressed as mean ± standard deviation, single-factor analysis of variance was used for comparison between multiple groups, and post hoc test (LSD) was used for comparison between groups. *t*-test was used for comparison between two groups. *P* < 0.05 indicates that the difference is statistically significant.

The article "The Levels of TNF-α, Tissue Factor, and Coagulation Function in Rats with Pulmonary Hypertension and the Intervention Effect of Sildenafil Encapsulated by Targeted Nanocarriers" was retracted in 2023. Reasons: unreliable results or conclusions; concerns about the data; concerns about the peer review; concerns about the citations.

## 3. Results and Discussion

### 3.1. The Levels of TNF-*α*, TF, and CF in Peripheral Blood of PAH Rats

As shown in Table 1 and Figure 1, the levels of TNF-*α*, TF, prothrombin time (PT), thrombin time (TT), and fibrinogen (FIB) levels in the peripheral blood of PAH rats were significantly higher than those of normal SD rat (*P* < 0.05).

### 3.2. Characterization of Targeted Nanocarriers Encapsulating Sildenafil

Nanoparticle size, PDI, and zeta potential are 194.32 ± 17.31 nm, 0.28 ± 0.02, and −6.34 ± 0.33, respectively. As shown in Figure 2, the sildenafil-containing nanoparticles have a complete shape and are almost spherical. The drug loading and encapsulation efficiency of nanoparticles were 24.61% and 70.52%, respectively.

### 3.3. In Vitro Drug Release from Carrier Nanoparticles

Figure 3 shows the drug release curves of drug-loaded nanoparticles in two physiological environments, pH 7.4 and pH 4.6. According to the 72 h cumulative drug release result, the drug-loaded nanoparticles completed the drug burst release within 12 h. At pH 7.4, the cumulative drug release amount of the drug-loaded nanoparticles was 42.18% at 12 hours, and the cumulative drug release rate reached 57.72% after 72 hours. At pH 4.6, the cumulative drug release amount for 12 hours was 55.32%, and after 72 hours, the cumulative drug release amount reached 65.23%. It shows that the release of the drug will not be affected under low pH conditions.

### 3.4. Intervention Effect of Targeted Nanocarrier Encapsulation Sildenafil on PAH Rats

As shown in Table 2 and Figure 4, compared with the normal rat group, the mean pulmonary artery pressure of the NS group, sildenafil group, TNC-E group, and CNC-sildenafil group was obviously increased; the media thickness of small pulmonary blood vessels increased obviously; the area of myocardial cells increased obviously. The levels of TNF-*α*, TF, and fibrinogen were obviously increased (*P* < 0.05). Compared with the NS group, the mean pulmonary artery pressure in the TNC-sildenafil group was obviously lower; the media thickness of small pulmonary blood vessels and the area of myocardial cells were obviously reduced; the levels of TNF-*α*, TF, and fibrinogen were obviously reduced (*P* < 0.05).

### 3.5. Discussion

Pulmonary hypertension (PAH) has a wide range of causes, and the pathogenesis of PAH is still unclear. Through literature survey, it is found that abnormally elevated CF will promote the occurrence and development of PAH, and inflammatory factors may play a dominant role in the change of CF [7, 8]. Therefore, this article explores the role of TNF-*α* and TF in the pathogenesis of pulmonary hypertension and the CF. Inflammation will promote the proliferation of pulmonary artery smooth muscle cells [16]. TNF-*α* can induce inflammation and promote granuloma formation and tissue fibrosis [17]. Related studies have found that the proliferation of pulmonary artery smooth muscle cells is related to the increase of TNF-*α* levels. Increased levels of TNF-*α* promote the remodeling of pulmonary blood vessels, leading to the occurrence of PAH [18]. The results of this study showed that the level of TNF-*α* in the peripheral blood of PAH rats was significantly higher than that of normal SD rats, further confirming that TNF-*α* promotes the occurrence and development of PAH.

The article "The Levels of TNF-α, Tissue Factor, and Coagulation Function in Rats with Pulmonary Hypertension and the Intervention Effect of Sildenafil Encapsulated by Targeted Nanocarriers" was retracted in 2023. Reasons: unreliable results or conclusions; concerns about the data; concerns about the peer review; concerns about the citations.

TF is the promoter of the exogenous coagulation pathway, and the exogenous coagulation pathway is the most critical link to initiate coagulation [19]. TF mainly exerts coagulation effect by combining with coagulation factor VII/VIIa. After it forms a complex with VIIa, it will accelerate the activation of coagulation factor X and can promote the conversion of coagulation factor X into Xa by activating coagulation factor IX. This series of mechanisms will lead to the production of thrombin [20]. TF distribution is tissue-specific: the content of extravascular components is higher. Under normal physiological conditions, the content of plasma TF is low, and cells in direct contact with blood do not express TF. Under pathological conditions, pathogenic factors can induce circulating monocytes to express TF, including factors such as tissue damage, malignant tumors, and cardiovascular diseases, which significantly increase the level of TF in blood circulation [21]. TF activated by protease receptors can cooperate with other coagulation factors to promote pleiotropic inflammatory response [22]. TF participates in the coagulation cascade, and the coagulation-inflammation crossreaction mediated by it is mutually activated and mutually promoted to form an inflammation-coagulation-thrombus cycle [23]. When PAH undergoes characteristic vascular remodeling, it is often accompanied by changes in blood hypercoagulability, but the mechanism is not yet clear. Studies have shown that the increased expression of TF is associated with blood hypercoagulability and pulmonary thrombosis [24, 25]. The results of this study showed that the levels of TF and CF in PAH rats were abnormally increased. It is suggested that increased expression of TF induces changes in CF, makes pulmonary artery blood in a hypercoagulable state, and promotes the occurrence and development of PAH.

Sildenafil is a drug for the clinical treatment of PAH, but the drug is not effective in improving the patient's activity endurance and long-term survival rate, which may be closely related to the drug's inability to achieve an effective therapeutic concentration in the lung tissue damaged blood vessel. GLUT-1 is upregulated in lung tissue and accelerates glucose transport. At the same time, the expression of GLUT-1 increased in the pulmonary vascular injury site of monocrotaline pulmonary hypertension rats and 18FD accumulated in the pulmonary blood vessels [14]. Studies have found that groups with a glucose-based target head can be actively taken up by GLUT-1 on the surface of the blood-brain barrier, which is conducive to drug transport to brain tissue [26]. Therefore, in this study, glucose-based modified nanocarriers were used to encapsulate sildenafil and compared with pure sildenafil on the effect of pulmonary hypertension. The results show that the targeted nanocarrier encapsulating sildenafil drug can significantly reduce the average pulmonary artery pressure, TNF-*α*, TF levels in PAH rats, restore the CF level to a normal state, and then improve the proliferation of small pulmonary blood vessels and media and right ventricular hypertrophy. Due to the strong affinity between the targeted nanocarrier and the target site, the drug can be effectively transported to the target tissue and effectively released, so that the drug concentration of the target tissue is increased, and the sildenafil can reach an effective therapeutic concentration in the lung tissue damaged blood vessel site. Lin et al. prepared PLGA-nanocarrier-encapsulated dictamnine (Dic-PLGA-NC), and they demonstrate that Dic-PLGA-NC efficiently penetrated the dermal layer, making it superior to naked dictamnine; moreover, it ameliorated the dermatitis symptoms and inflammatory cytokine expression in vivo [27]. Consistent with the results of this study, PLGA-nanocarrier has the effect of targeted drug delivery. Makled et al. prepared solid lipid nanoparticles (SLNs) loaded with sildenafil citrate, and they demonstrate that SLNs has the potential of a pulmonary drug delivery system and might give promises of new therapy for pH of higher safety, better performance, and higher patient compliance [28]. The results of this study prove that targeting nanocarrier encapsulation of sildenafil can obviously reduce the average pulmonary artery pressure in rats with pulmonary hypertension, improve pulmonary vascular media proliferation and myocardial hypertrophy, and restore the levels of TNF-*α*, TF, and CF to a normal state. Targeting nanocarrier encapsulation of sildenafil may have higher performance in the treatment of pulmonary hypertension. This study indicated the feasibility of targeted nanocarriers as localized delivery of sildenafil to the lung. However, the treatment of targeted nanocarriers to encapsulate sildenafil is still questionable. Most of the experiments are conducted in animals (rats, dogs, and lambs), and its effect on human beings still needs further discussion.

The article "The Levels of TNF-α, Tissue Factor, and Coagulation Function in Rats with Pulmonary Hypertension and the Intervention Effect of Sildenafil Encapsulated by Targeted Nanocarriers" was retracted in 2023. Reasons: unreliable results or conclusions; concerns about the data; concerns about the peer review; concerns about the citations.

## 4. Conclusion

In this study, the monocrotaline-induced rat pulmonary hypertension (PAH) model was constructed. After detecting the levels of TNF-*α*, TF, and CF in the peripheral blood of PAH rats, it was found that the levels of TNF-*α*, TF, and CF were abnormally elevated. It is suggested that the levels of TNF-*α*, TF, and CF are significantly related to the occurrence and development of PAH. In order to explore drugs with significant curative effects on PAH rats, we prepared targeted nanocarriers to encapsulate sildenafil. The drug-loaded particles can obviously reduce the average pulmonary artery pressure in PAH rats and improve the proliferation of small pulmonary blood vessels and the myocardial hypertrophy. The mechanism may be to effectively reduce the levels of TNF-*α* and TF to restore the CF level to a normal state, thereby improving the symptoms of PAH rats.

## Figures and Tables

**Figure 1:** Comparison of peripheral blood TNF-*α*, tissue factor, and coagulation function between PAH rats and normal rats. (a) Mean pulmonary artery pressure. (b) TNF-*α* level in peripheral blood. (c) Tissue factor level. (d) Prothrombin time (PT). (e) Thrombin time (TT). (f) Fibrinogen (FIB) level. ^∗∗∗^*P* < 0.001, comparison between two groups.

**Figure 2:** Transmission electron microscope image of nanoparticles containing sildenafil.

**Figure 3:** In vitro drug release curves of sildenafil-loaded nanoparticles under different pH conditions.

**Figure 4:** The therapeutic effect of targeted nanocarrier encapsulation sildenafil on PAH rats. (a) Mean pulmonary artery pressure (mmHg). (b) Media thickness of small pulmonary blood vessels (%). (c) Cardiomyocyte area (*μ*m^2^). (d) Tumor necrosis factor-*α* (ng/L). (e) Tissue factor (pg/mL). (f) Fibrinogen (g/L).

**Table 1:** Peripheral blood TNF-*α*, tissue factor, and coagulation function levels in PAH rats.

	Mean pulmonary artery pressure (mmHg)	TNF-*α* (ng/L)	Tissue factor (pg/mL)	Prothrombin time (s)	Thrombin time (s)	Fibrinogen (g/L)
Normal SD rats (*n* = 6)	18.62 ± 1.67	0.18 ± 0.04	25.80 ± 2.99	8.54 ± 1.13	40.41 ± 1.67	1.82 ± 0.37
PAH rats (*n* = 6)	35.93 ± 2.11	1.67 ± 0.30	43.83 ± 4.23	16.64 ± 2.33	62.68 ± 4.12	4.49 ± 0.74
*t*	15.710	12.195	8.500	7.649	12.246	7.902
*P*	<0.001	<0.001	<0.001	<0.001	<0.001	<0.001

**Table 2:** Intervention effect of targeted nanocarrier encapsulation sildenafil on PAH rats.

Group	Mean pulmonary artery pressure (mmHg)	Pulmonary small blood vessel media thickness (%)	Cardiac cell area (*μ*m^2^)	TNF-*α* (ng/L)	Tissue factor (pg/mL)	Fibrinogen (g/L)
Normal SD rat (*n* = 6)	18.62 ± 1.67	34.30 ± 1.24	174.21 ± 11.60	0.18 ± 0.04	25.80 ± 2.99	1.82 ± 0.37
NS group (*n* = 6)	35.74 ± 2.10^a^	60.55 ± 3.16^a^	339.44 ± 21.37^a^	1.66 ± 0.30^a^	42.95 ± 4.45^a^	4.35 ± 0.69^a^
Sildenafil group (*n* = 6)	29.09 ± 1.86^a^	57.41 ± 3.02^a^	309.88 ± 24.00^a^	1.37 ± 0.29^a^	36.68 ± 4.03^a^	3.71 ± 0.46^a^
TNC-E group (*n* = 6)	35.15 ± 2.30^a^	60.40 ± 3.47^a^	339.72 ± 22.80^a^	1.60 ± 0.29^a^	41.41 ± 3.91^a^	4.21 ± 0.59^a^
CNC-sildenafil group (*n* = 6)	28.90 ± 1.98^a^	55.51 ± 2.82^a^	289.39 ± 21.07^a^	1.21 ± 0.20^a^	37.09 ± 3.87^a^	3.61 ± 0.50^a^
TNC-sildenafil group (*n* = 6)	23.71 ± 2.01^b^	40.79 ± 2.52^b^	193.05 ± 19.00^b^	0.50 ± 0.08^b^	27.90 ± 2.99^b^	2.46 ± 0.40^b^
*F*	65.892	95.046	76.931	42.419	20.970	22.133
*P*	<0.001	<0.001	<0.001	<0.001	<0.001	<0.001

Note: ^a^ means *P* < 0.05 compared with normal SD rats. ^b^ means *P* < 0.05 compared with the NS group. NS group: normal saline; sildenafil group: sildenafil; TNC-E group: targeted nanoempty carrier: CNC-sildenafil group: ordinary nanocarrier encapsulated sildenafil; TNC-sildenafil group: targeted nanocarrier encapsulation sildenafil.

The article "The Levels of TNF-α, Tissue Factor, and Coagulation Function in Rats with Pulmonary Hypertension and the Intervention Effect of Sildenafil Encapsulated by Targeted Nanocarriers" was retracted in 2023. Reasons: unreliable results or conclusions; concerns about the data; concerns about the peer review; concerns about the citations.

## Data Availability

The labeled dataset used to support the findings of this study are available from the corresponding author upon request.
